The article "A Traceable Blockchain-Based Vaccination Record Storage and Sharing System" was published in 2022. Journal: J Healthc Eng.

# A Traceable Blockchain-Based Vaccination Record Storage and Sharing System

**DOI:** 10.1155/2022/2211065

**Published:** 2022-03-09

**Authors:** Jingshou Chen, Xiaofeng Chen, Chin-Ling Chen

**Affiliations:** ^1^Department of Infectious Diseases, The First Affiliated Hospital of Xiamen University, Xiamen 361003, China; ^2^School of Electronic Information Science, Fujian Jiangxia University, Fuzhou 35010, China; ^3^School of Information Engineering, Changchun Sci-Tech University, Changchun 130600, China; ^4^School of Computer and Information Engineering, Xiamen University of Technology, Xiamen 361024, China; ^5^Department of Computer Science and Information Engineering, Chaoyang University of Technology, Taichung 41349, Taiwan

## Abstract

Blockchain technology is essentially a decentralized database maintained by relevant parties and has been widely used in various scenarios such as logistics and finance. In terms of applications in the medical field, it is becoming more and more important because the patient's symptoms may be related to a certain vaccine. Whether the patient has been vaccinated with this vaccine will lead to different diagnostic results by the doctor. However, in the current vaccination environment of many regions, the vaccination record (VR) can only be kept in the patient's vaccination booklet, which is easy to lose or destroy. Therefore, the doctor needs to retrieve the patient's VR through a centralized database maintained by the government, which is time-consuming and will increase the medical risk. This study proposes a traceable blockchain-based vaccination record storage and sharing system. In the proposed system, the patient gets the vaccination at any legal clinic and the VR can be saved accompanied by the signature into the blockchain center, which ensures traceability. When the patient visits the hospital for treatment, the doctor can obtain the detail of the VR from the blockchain center and then make a diagnosis. The security of the proposed system will be protected by the programmed smart contracts. Through mutual authentication, our system can also provide and guarantee data integrity and nonrepudiation. Moreover, the proposed system has resistance to replay and man-in-the-middle attacks, and the performance is good.

## 1. Introduction

The rapid evolution of information technology is giving more convenience to our daily lives. Electronic health records (EHRs), including medical payment records, medical treatment records, and medical history, are gathered and stored in the private servers of the hospitals [1–5] and now is drawing increasing attention as it contains personal privacy information. For multiple reasons including to improve the quality of services, the traditional paper-based systems have been replaced by the electronic health system for storing and processing EHRs based on a more flexible, more efficient, and more convenient platform.

The article "A Traceable Blockchain-Based Vaccination Record Storage and Sharing System" was published in 2022. Journal: J Healthc Eng.

It should be noticed that nowadays in many regions, vaccination recording is still in a traditional way that is not keeping up with developing technologies. The patient can only be vaccinated in a clinic nearby with a vaccine booklet that records the vaccination. The detail of the vaccination record (VR) is stored in the clinic and will be uploaded into a centralized database maintained by the government. Without the vaccine booklet, the patient cannot tell what vaccine he/she has gotten, not to mention the vaccination time and the detailed information of the vaccination phase. Unfortunately, the vaccine booklet has vulnerability to forgery, alteration, and loss. Furthermore, under the current vaccination system, the patient's VR is not directly shared between the clinic and the hospital. When the patient visits the hospital for treatment of a symptom without the vaccine booklet, and the symptom is related to a certain vaccine (for example, varicella-zoster virus), the hospital cannot directly gain the VR from the clinic but needs to retrieve it through the centralized database. The retrieving phase is very time-consuming and will increase the medical risk [6–10]. Therefore, allowing the patients and the doctors to track and retrieve the VR at any time is an important issue that needs to be resolved in the current stage of research.

Meanwhile, the vaccination records (VRs) need to be carefully protected as important privacy information. The centralized database provides a controlled and easy-access solution for maintaining the VRs. However, the security of VRs is bound to be threatened when the failure occurs in the centralized database. Besides, decentralized databases offer another solution for data protection. Compared with the centralized database, the data in the decentralized database are scattered and stored in different places. The collapse of one database will not lead to the failure of all the decentralized databases, so the decentralized databases have better security than the centralized database.

How to provide flexible data sharing is another concern in VRs. Centralized databases store the VRs in one place. Although this is convenient for data management, it virtually imposes a heavy burden on the server. As a result, it is not conducive to rapidly sharing the VRs via centralized databases. Decentralized databases can access its different separated databases through different channels, so they can provide efficient VR sharing.

The article "A Traceable Blockchain-Based Vaccination Record Storage and Sharing System" was published in 2022. Journal: J Healthc Eng.

Blockchain technology is essentially a decentralized database collectively maintained and has been widely employed in various fields [11–15]. As there is no need for third-party trust endorsements, blockchain can create a fully trusted environment between unfamiliar involved parties. Furthermore, it can ensure traceability, irreparable modification, nonrepudiation, and privacy protection through cryptography technology. Therefore, blockchain technology has been seen as a powerful tool to address the above problems in current vaccination recording systems through its attractive features.

Based on the foregoing overview, a blockchain-based vaccination record storage and sharing system is proposed, to provide traceable VRs and support the data sharing of confidential VRs. In our proposed system, the detail of the VR with the signature will be permanently stored in the blockchain center after the vaccination, thereby ensuring the integrity of the data.

In detail, the contributions of our study are listed below.

1. Each role in our blockchain-based vaccination record storage and sharing system is specifically defined. In our method, the traceability and the integrity of VR are guaranteed by blockchain technology.
2. BAN logic is used to identify the identity to provide communication security between two parties.
3. Through the characteristics of the blockchain, our system can resist a variety of attacks, i.e., replay attack and man-in-the-middle attack. Meanwhile, the performance of our system is elaborated by the computation cost, communication cost analysis, and functionality comparison.

The rest of this study is organized as follows.  Section 2 reviews related work. In Section 3, the preliminary and security requirements of the proposed system will be briefly introduced. The proposed vaccination record storage and sharing system is described in a detailed way in Section 4.  Section 5 and Section 6 show the security and performance analysis of the proposed system, respectively.  Section 7 presents our conclusions.

## 2. Related Works

The massive growth of medical data impels traditional medical data management schemes to expose the defects. To overcome the drawbacks and improve the medical services, some medical systems have been proposed [16–24]. The medical systems applying cloud computing have already shown good performance in storing and processing the EHRs between different medical institutions [16, 17]. However, on the one hand, the current cloud-based systems have no superiority in privacy protection for the EHRs; on the other hand, these systems have not achieved a satisfactory data sharing mechanism. Thus, Xia et al. [18] proposed a blockchain-based system for the effective management and protection of medical records in 2017. The security of the storage data is guaranteed by authenticating user identities and using encryption mechanisms. However, the system had the risk of data leakage during the data sharing process, making the system unsuitable for real-world applications. Zheng et al. [19] designed a medical data sharing scheme that combines blockchain and cloud computing. Their scheme realized the sharing of medical data between participating parties. However, the data receiver does not know the correctness of the received data since the integrity of the received medical data cannot be verified. Xia et al. [20] introduced an electronic medical record sharing scheme based on blockchain. The tamper-resistant feature of the blockchain technology is used in their method to ensure the security of the medical records. However, the patient cannot track their EHRs in real time. Later, Yang et al. [21] suggested a blockchain-based EHR system. Although their system has good compatibility with some existing systems, their system is not efficient because the creation and verification of new blocks are all handled by a single party.

The article "A Traceable Blockchain-Based Vaccination Record Storage and Sharing System" was published in 2022. Journal: J Healthc Eng.

Although some secure medical systems based on electronic medical records (EMRs) have been proposed in the past, there is not much research on the medical system based on VRs [25–28]. In 2021, Hofstetter et al. [25] introduced a strategy to offer vaccinations in nonprimary care settings such as schools, hospitals, and pharmacies. However, their method can only be used to solve the restriction in the specific clinic. An electronic vaccination certificate (EVC) is developed to replace traditional vaccination record booklets. Yet, EVC is mainly used to record COVID-19 vaccination. Eisenstadt et al. [26] used the EVC as “Immunity Passport” for COVID-19. They designed a smartphone app that connects to a centralized database that can store patients' vaccination status. Based on that record, the app generates a token or QR (“quick response”) code signifying the vaccination status, which can then be verified by authorized parties. The EVC faces two significant challenges: interoperability and privacy [28]. Since the EVC standards established in different places are not uniform, how to realize cross-regional EVC recognition is important for the broad and easy usability of digital vaccination certificates. Data privacy is important for user trust and legal compliance making it the de facto crucial challenge than interoperability.

Based on the existing analysis of research scholars, it is foreseeable that the service quality of the medical systems can be further facilitated with the combination of blockchain technology. On the other side, it cannot be ignored that blockchain-based medical systems still have flaws in the privacy protection of data storage and sharing. Particularly, the electrification of VRs is still under development. How to allow patients to track and grasp their VRs meanwhile realizing the sharing of vaccine records between different institutions is an urgent problem to be solved. These issues are exactly the concerns of this study. In our proposed traceable blockchain-based vaccination record storage and sharing system, every VR is stored in the blockchain through the smart contract and granted secure data sharing in the future. It is visible that our scheme shows the way to fill the gaps of existing research.

The article "A Traceable Blockchain-Based Vaccination Record Storage and Sharing System" was published in 2022. Journal: J Healthc Eng.

## 3. Preliminary and Security Requirements

In this section, the preliminary requirements, including the BAN logic, ECDSA, and the smart contract, are elaborated in subsection 3.1.  Subsection 3.2 shows the security requirements of the proposed scheme.

### 3.1. Preliminary

#### 3.1.1. BAN Logic

The Burrows-Abadi-Needham (BAN) logic proof model [29] is widely applied in security-related scholars for proving whether the mutual authentication has been achieved of a protocol or scheme.

#### 3.1.2. ECDSA

To guarantee the security of the transmitted and exchanged message in the digital network, several encryption systems have been proposed by scholars. The elliptic curve digital signature algorithm (ECDSA), derived from the digital signature algorithm (DSA) [30], involves the concept of elliptic curve cryptography (ECC) [31]. While compared to DSA, the ECC reduces the key size in the algorithm and also provides a faster calculation speed.

#### 3.1.3. Smart Contract

The smart contract [32] is a computer protocol designed to spread, verify, and execute a contract in a digital form. The promised agreement between each contract participant can be executed on it. The collaboration and trust between each contract participant can be achieved in blockchain through smart contracts, which can expand the cooperation between each party.

With the development of medical technology, a large amount of information about patients' vaccination records, medical histories, and medical payment records needs to be reserved. These records are not only stored in the local server but also permanently conserved in the blockchain by the smart contracts. When a patient visits different medical institutions, he/she can authorize medical staff to retrieve the history VR from the BC through the smart contract. Thus, the medical staff can provide better health services with the help of historical medical records.

The article "A Traceable Blockchain-Based Vaccination Record Storage and Sharing System" was published in 2022. Journal: J Healthc Eng.

### 3.2. Security Requirements

The security requirements of our vaccination record storage and sharing system are listed as follows.

1. Mutual authentication: in a proposed system, each party must confirm the legal identity of other parties in every phase. If any two parties can confirm one another's legal identity, then mutual authentication is achieved.
2. Data integrity: in an insecure network environment, the message delivered from the sender may be modified by a malicious attacker. Thus, the integrity of the transferred message must be maintained and should be ensured that it can defend against tampering during the transmission.
3. Nonrepudiation: in each information exchange phase, the sender cannot refuse to acknowledge that the message he has been sent. A secure system must achieve nonrepudiation requirements.
4. Resisting replay attacks: the communication between two parties may be intervened by malicious attackers. The malicious attackers will pretend to be a legitimate sender and send identical information to the intended receiver. This situation will lead to the leak of personal data security and, therefore, must be prevented.
5. Resisting man-in-the-middle attacks: the attacker may intercept the message communicated between the sender and the receiver, and then, he/she can obtain the content of the message in the middle. This situation must be prevented too.

## 4. Proposed Scheme

In this section, we introduce the construction and workflow of our system in detail. The system framework is shown first. Then, the meaning of some notations is elaborated as follows.

### 4.1. System Framework

This study proposes a blockchain-based vaccination record storage and sharing system.  Figure 1 shows the main architecture of the proposed system, which is composed of four parties, including the blockchain center, the patient, the clinic, and the hospital. The detail of each party is described below.

1. Blockchain center (BC) : The blockchain center is owned by the government. It manages all relevant data and operations on personal mobile devices and medical devices of the clinics and the hospitals. All mobile devices and medical devices need to be registered in the BC, and then, the three parties can mutually authenticate each other.
2. Patient: Each patient carries a personal mobile device with them. The device stores a verification message that can uniquely identify the patient. Moreover, the primary message of the VR will be reserved in the personal mobile device and will be provided to the hospital in the future to diagnose.
3. Clinic: The patient will be vaccinated at the clinic. The doctor of the clinic uses a medical device that can uniquely identify the clinic. When the patient goes to the clinic for vaccination, the doctor of the clinic can execute the vaccination for the patient and store the VR into the BC. Also, the patient will store the primary message of the VR on his/her mobile device.
4. Hospital: The patient will be diagnosed in the hospital. The doctor of the hospital uses a medical device that can uniquely identify the hospital's identification. When the patient goes to the hospital seeking treatment for a symptom, the doctor of the hospital can retrieve the VRs through the primary message of the VR stored in the patient mobile device and further provide the diagnosis for the patient.

The article "A Traceable Blockchain-Based Vaccination Record Storage and Sharing System" was published in 2022. Journal: J Healthc Eng.

The following is a description of our method. It should be noticed that all parties must register their corresponding devices in the BC and retrieve a unique ID and a private and public key pair from BC, respectively.

  Step 1: The patient goes to the clinic with his/her mobile device for vaccination, and the clinic and the patient must authenticate one another's identity first. After mutual authentication, the doctor of the clinic will carry out the vaccination for the patient.
  Step 2: The doctor of the clinic will save the VR in the local server of the clinic and store VR into the BC through the smart contract technology.
  Step 3: The BC feedbacks the storage result to the clinic.
  Step 4: The doctor of the clinic returns the primary message of the VR to the patient, and the patient saves the message on his/her mobile device.
  Step 5: The patient visits the hospital with his/her mobile device for treatment of a symptom, and the hospital and the patient must also authenticate each other identity first. After mutual authentication, the patient provides the VR history in his mobile device to the doctor.
  Step 6: The doctor of the hospital retrieves the VRs from the BC according to the information acquired from the patient.
  Step 7: The BC feedbacks the details of VRs to the hospital.
  Step 8: The doctor of the hospital provides the diagnostic results for the patient based on the VRs.

### 4.2. Notations

The notations used in the study are listed in Table 1.

### 4.3. Initialization Phase

The fundamental chaincode structure of the proposed scheme is elaborated in this section.  Figure 2 shows the information structure of the access parties (APs) and the enumeration of the role type.  Figure 3 shows the structure to store the vaccination record in the BC.

### 4.4. Registration Phase

All parties need to register from the BC. The BC generates and sends the identity, public, and private key pair to the parties. The main process of the registration is presented as shown in Figure 4.

The article "A Traceable Blockchain-Based Vaccination Record Storage and Sharing System" was published in 2022. Journal: J Healthc Eng.

**Step 1 .**

The access party (AP) provides the primary information (i.e., name and role) and sends a registration request to the BC.

**Step 2 .**

The BC generates an ECDSA private key *d*_*X*_ and calculates public key *Q*_*X*_ by the following:

(1) $$\begin{array}{c} Q_{X}=d_{X}G. \end{array}$$

The information provided by the AP needs to be validated by the BC. If it is valid, the algorithm “Registration” will be executed, as shown in Algorithm 1. Then, BC sends (*ID*_*X*_, *d*_*X*_, *Q*_*X*_) to AP.

**Step 3 .**

AP stores (*ID*_*X*_, *d*_*X*_, *Q*_*X*_) for signing the signature message.

### 4.5. Authentication Phase

In this phase, we define the “Sign” and “Verify” functions that implement the ECDSA to achieve identity authentication between User A and User B. The definitions of these two functions are shown in Algorithm 2 and Algorithm 3. When User A and User B exchange messages, the sender generates a signature with a “Sign” function to the receiver. When the receiver receives the message, they execute a “Verify” function to verify. The flowchart of the authentication phase is shown in Figure 5.

**Step 4 .**

User A selects a random number *R*_1_ and calculates *M*_*A*_ by equation (2). Then, User A calculates *h*_*A*_ by equation (3).

(2) $$\begin{array}{c} M_{A}=\left(ID_{A}||ID_{B}||T_{1}\right), \end{array}$$

(3) $$\begin{array}{c} h_{A}=H\left(M_{A}\right). \end{array}$$

The signatures are generated by executing the function “Sign” in Algorithm 2. In detail, User A calculates the parameters of ECDSA by equation (4) and generates the signatures by equations (5) and (6). Then, User A encrypted *M*_*A*_ with User B's public key by equation (7) and sends (*ID*_*A*_, *ID*_*B*_, *C*_*A*_, (*r*_*A*_, *s*_*A*_)) to User B.

(4) $$\begin{array}{c} \left(x_{A},y_{A}\right)=R_{1}G, \end{array}$$

(5) $$\begin{array}{c} r_{A}=x_{A}\mathrm{mod}n, \end{array}$$

(6) $$\begin{array}{c} s_{A}=x_{A}^{-1}\left(h_{A}+r_{A}d_{A}\right)\mathrm{mod}n, \end{array}$$

(7) $$\begin{array}{c} C_{A}=E_{PK_{B}}\left(M_{A}\right). \end{array}$$

**Step 5 .**

User B receives the message at *T*_2_ and decrypts *C*_*A*_ with its private key by the following:

(8) $$\begin{array}{c} M_{A}=D_{SK_{B}}\left(C_{A}\right). \end{array}$$

Then, User B validates the timestamp by

(9) $$\begin{array}{c} \left(T_{2}-T_{1}\right)\leq \tau ?. \end{array}$$

If it is valid, User B executes the function “Verify” in Algorithm 3 to validate the signature of User A. In detail, User B calculates the parameters by equations (10)–(13) and validates the signatures by equation (14).

(10) $$\begin{array}{c} h_{A}^{\prime }=H\left(M_{A}\right), \end{array}$$

(11) $$\begin{array}{c} u_{1}=h_{A}^{\prime }s_{A}^{-1}\text{mod }n, \end{array}$$

(12) $$\begin{array}{c} u_{2}=r_{A}s_{A}^{-1}\text{mod }n, \end{array}$$

(13) $$\begin{array}{c} \left(x_{A}^{\prime },y_{A}^{\prime }\right)=u_{1}G+u_{2}Q_{A}, \end{array}$$

(14) $$\begin{array}{c} x_{A}^{\prime }\overset{?}{=}r_{A}\text{ mod }n. \end{array}$$

If it is valid, User B selects a random number *R*_2_ and calculates *M*_*B*_ by equation (15). Then, User B calculates *h*_*B*_ by equation (16).

(15) $$\begin{array}{c} M_{B}=\left(ID_{A}||ID_{A}||T_{3}\right), \end{array}$$

(16) $$\begin{array}{c} h_{B}=H\left(M_{B}\right). \end{array}$$

The signatures are generated by executing the function “Sign” in Algorithm 2. In detail, User B calculates the parameters of ECDSA by equation (17) and generates the signatures by equations (18) and (19). Then, User B encrypted *M*_*B*_ with User A's public key by equation (20) and sends (*ID*_*B*_, *ID*_*A*_, *C*_*B*_, (*r*_*B*_, *s*_*B*_)) to User A.

(17) $$\begin{array}{c} \left(x_{B},y_{B}\right)=R_{2}G, \end{array}$$

(18) $$\begin{array}{c} r_{B}=x_{B}\mathrm{mod}n, \end{array}$$

(19) $$\begin{array}{c} s_{B}=x_{B}^{-1}\left(h_{B}+r_{B}d_{B}\right)\mathrm{mod}n, \end{array}$$

(20) $$\begin{array}{c} C_{B}=E_{PK_{A}}\left(M_{B}\right). \end{array}$$

**Step 6 .**

The article "A Traceable Blockchain-Based Vaccination Record Storage and Sharing System" was published in 2022. Journal: J Healthc Eng.

User A receives the message at *T*_4_ and decrypts *C*_*B*_ with its private key by the following:

(21) $$\begin{array}{c} M_{B}=D_{SK_{A}}\left(C_{B}\right). \end{array}$$

Then, User A validates the timestamp by the following:

(22) $$\begin{array}{c} \left(T_{4}-T_{3}\right)\leq \tau ?. \end{array}$$

If it is valid, User A executes the function “Verify” in Algorithm 3 to validate the signature of User B. In detail, User A calculates the parameters by equations (23)–(26) and validates the signatures by equation (27).

(23) $$\begin{array}{c} h_{B}^{\prime }=H\left(M_{B}\right), \end{array}$$

(24) $$\begin{array}{c} u_{1}=h_{B}^{\prime }s_{B}^{-1}\text{ mod }n, \end{array}$$

(25) $$\begin{array}{c} u_{2}=r_{B}s_{B}^{-1}\text{ mod }n, \end{array}$$

(26) $$\begin{array}{c} \left(x_{B}^{\prime },y_{B}^{\prime }\right)=u_{1}G+u_{2}Q_{B}, \end{array}$$

(27) $$\begin{array}{c} x_{B}^{\prime }\overset{?}{=}r_{B}\text{ mod }n. \end{array}$$

### 4.6. Patient Vaccination Phase

The patient can visit any clinic that has registered in BC for vaccination. After the mutual authentication, the patient issues the clinic the name of the vaccination and gets the vaccination. The vaccine record will be saved in the mobile device of the patient and the local server of the clinic. Meanwhile, the signature of the patient and the clinic, and the hash value of the record accompanied by the identities of the patient, clinic, and vaccine will be stored in BC. The patient vaccination phase consists of five steps, as shown in Figure 6. The detail of each step is described below.

The article "A Traceable Blockchain-Based Vaccination Record Storage and Sharing System" was published in 2022. Journal: J Healthc Eng.

**Step 7 .**

The patient selects a random number *R*_3_ and calculates *M*_*P*_ with the name of the vaccination, *V*, by equation (28). Then, the patient calculates *h*_*P*_ by equation (29).

(28) $$\begin{array}{c} M_{P}=\left(ID_{P}||ID_{C}||V||T_{5}\right), \end{array}$$

(29) $$\begin{array}{c} h_{P}=H\left(M_{P}\right). \end{array}$$

The signatures (*r*_*P*_, *s*_*P*_) are generated by executing the function “Sign” in Algorithm 2, as shown in the following:

(30) $$\begin{array}{c} \left(r_{P},s_{P}\right)=Sign\left(h_{P},R_{3},d_{P}\right). \end{array}$$

Then, the patient encrypted *M*_*P*_ with the public key of the clinic by equation (31) and sends (*ID*_*P*_, *ID*_*C*_, *C*_*P*_, (*r*_*P*_, *s*_*P*_)) to the clinic.

(31) $$\begin{array}{c} C_{P}=E_{PK_{C}}\left(M_{P}\right). \end{array}$$

**Step 8 .**

The clinic receives the message at *T*_6_ and decrypts *C*_*P*_ with its private key by the following:

(32) $$\begin{array}{c} M_{P}=D_{SK_{C}}\left(C_{P}\right). \end{array}$$

Then, the clinic validates the timestamp by the following:

(33) $$\begin{array}{c} \left(T_{6}-T_{5}\right)\leq \tau ?. \end{array}$$

If it is valid, the clinic calculates *h*_*P*_′ and executes the function “Verify” in Algorithm 3 to validate the signature of the patient by equations (34) and (35).

(34) $$\begin{array}{c} h_{P}^{\prime }=H\left(M_{P}\right), \end{array}$$

(35) $$\begin{array}{c} \mathrm{Verify}\left(h_{P}^{\prime },r_{P},s_{P}\right). \end{array}$$

If the signature is valid, the clinic executes the vaccination for the patient and generates the vaccination record, *VR*, including *ID*_*P*_, *ID*_*V*_ (the identity of the vaccination *V*), *ID*_*C*_, the time of the vaccination, and other detailed information. At the same time, the primary message of *VR*, denoted as *K*_*VR*_, is generated and delivered to the patient.

Next, the clinic selects a random number *R*_4_ and calculates *M*_*C*_ with *VR* by equation (36). Then, the clinic calculates *h*_*C*_ by equation (37).

(36) $$\begin{array}{c} M_{C}=\left(ID_{C}||ID_{P}||K_{VR}||T_{7}\right), \end{array}$$

(37) $$\begin{array}{c} h_{C}=H\left(M_{C}\right). \end{array}$$

The signatures (*r*_*C*_, *s*_*C*_) are generated by executing the function “Sign” in Algorithm 2, as shown in the following:

(38) $$\begin{array}{c} \left(r_{C},s_{C}\right)=Sign\left(h_{C},R_{4},d_{C}\right). \end{array}$$

The algorithm “RIns” is triggered to create a record stored in BC, the algorithm of which is shown in Algorithm 4. The record includes the signature of the patient and the clinic.

The article "A Traceable Blockchain-Based Vaccination Record Storage and Sharing System" was published in 2022. Journal: J Healthc Eng.

Finally, the clinic encrypted *M*_*C*_ by the public key of the patient by equation (39) and sends (*ID*_*C*_, *ID*_*P*_, *C*_*C*_, (*r*_*C*_, *s*_*C*_)) to the patient.

(39) $$\begin{array}{c} C_{C}=E_{PK_{H}}\left(M_{C}\right). \end{array}$$

**Step 9 .**

The patient receives the message at *T*_8_ and decrypts *C*_*C*_ with its private key by the following:

(40) $$\begin{array}{c} M_{C}=D_{SK_{P}}\left(C_{C}\right). \end{array}$$

Then, the patient validates the timestamp by the following:

(41) $$\begin{array}{c} \left(T_{8}-T_{7}\right)\leq \tau ?. \end{array}$$

If it is valid, the patient calculates and executes the function “Verify” in Algorithm 3 to validate the signature of the clinic by equations (42) and (43).

(42) $$\begin{array}{c} h_{C}^{\prime }=H\left(M_{C}\right), \end{array}$$

(43) $$\begin{array}{c} \mathrm{Verify}\left(h_{C}^{\prime },r_{C},s_{C}\right). \end{array}$$

If the signature is valid, the patient stores the *K*_*VR*_ on his/her mobile device.

### 4.7. Patient Treatment Phase

When the patient visits the hospital for treatment of a symptom related to vaccination history, mutual authentication should be first executed. After the authentication, the hospital will obtain the VR from BC by *K*_*VR*_, which is stored in a patient mobile device. After verifying the record with the hash value, the hospital performs a diagnosis and issues the diagnostic result about the patient. The patient treatment phase consists of five steps, as shown in Figure 7. The detail of each step is described below.

**Step 10 .**

The patient selects a random number *R*_5_ and calculates *M*_*P*2_ with the symptom, *S*, by equation (44). Then, the patient calculates *h*_*P*2_ by equation (45).

(44) $$\begin{array}{c} M_{P2}=\left(ID_{P}||ID_{H}||S||K_{VR}||T_{9}\right), \end{array}$$

(45) $$\begin{array}{c} h_{P2}=H\left(M_{P2}\right). \end{array}$$

The signatures (*r*_*P*2_, *s*_*P*2_) are generated by executing the function “Sign” in Algorithm 2, as shown in the following:

(46) $$\begin{array}{c} \left(r_{P2},s_{P2}\right)=Sign\left(h_{P2},R_{5},d_{P}\right). \end{array}$$

Then, the patient encrypted *M*_*P*2_ with the public key of the hospital by equation (47) and sends (*ID*_*P*_, *ID*_*H*_, *C*_*P*2_, (*r*_*P*2_, *s*_*P*2_)) to the hospital.

(47) $$\begin{array}{c} C_{P2}=E_{PK_{H}}\left(M_{P2}\right). \end{array}$$

**Step 11 .**

The hospital receives the message at *T*_10_ and decrypts *C*_*P*2_ with its private key by the following:

(48) $$\begin{array}{c} M_{P2}=D_{SK_{H}}\left(C_{P2}\right). \end{array}$$

Then, the hospital validates the timestamp by the following:

(49) $$\begin{array}{c} \left(T_{10}-T_{9}\right)\leq \tau ?. \end{array}$$

If it is valid, the hospital calculates and executes the function “Verify” in Algorithm 3 to validate the signature of the patient by equations (50) and (51).

(50) $$\begin{array}{c} h_{P2}^{\prime }=H\left(M_{P2}\right), \end{array}$$

(51) $$\begin{array}{c} \mathrm{Verify}\left(h_{P2}^{\prime },r_{P2},s_{P2}\right). \end{array}$$

If the signature is valid, the algorithm “RGet” is triggered to retrieve the *VR*. The definition of “RGet” is shown in Algorithm 5. Since the records contain the signatures of the patients and the clinics, it is convenient to track the validation of the record.

The article "A Traceable Blockchain-Based Vaccination Record Storage and Sharing System" was published in 2022. Journal: J Healthc Eng.

Next, the hospital selects a random number *R*_6_ and calculates *M*_*H*_ with the diagnostic result of the patient, *D*, by equation (52). Then, the hospital calculates *h*_*H*_ by equation (53).

(52) $$\begin{array}{c} M_{H}=\left(ID_{H}||ID_{P}||D||T_{11}\right), \end{array}$$

(53) $$\begin{array}{c} h_{H}=H\left(M_{H}\right). \end{array}$$

The signatures (*r*_*H*_, *s*_*H*_) are generated by executing the function “Sign” in Algorithm 2, as shown in the following:

(54) $$\begin{array}{c} \left(r_{H},s_{H}\right)=Sign\left(h_{H},R_{6},d_{H}\right). \end{array}$$

Finally, the hospital encrypted *M*_*H*_ by the public key of the patient by equation (55) and sends (*ID*_*H*_, *ID*_*P*_, *C*_*H*_, (*r*_*H*_, *s*_*H*_)) to the patient.

(55) $$\begin{array}{c} C_{H}=E_{PK_{P}}\left(M_{H}\right). \end{array}$$

**Step 12 .**

The patient receives the message at *T*_12_ and decrypts *C*_*H*_ with its private key by the following:

(56) $$\begin{array}{c} M_{H}=D_{SK_{P}}\left(C_{H}\right). \end{array}$$

Then, the patient validates the timestamp by the following:

(57) $$\begin{array}{c} \left(T_{12}-T_{11}\right)\leq \tau ?. \end{array}$$

If it is valid, the patient calculates and executes the function “Verify” in Algorithm 3 to validate the signature of the hospital by equations (58) and (59).

(58) $$\begin{array}{c} h_{H}^{\prime }=H\left(M_{H}\right), \end{array}$$

(59) $$\begin{array}{c} \mathrm{Verify}\left(h_{H}^{\prime },r_{H},s_{H}\right). \end{array}$$

If the signature is valid, the patient stores the *D* in his/her mobile device.

## 5. Security Analysis

We will analyze the security of our system in terms of the following aspects.

### 5.1. Mutual Authentication

In this section, we use the BAN logic proof model to prove that mutual authentication in the authentication phase is guaranteed in our proposed system. The common notations used in the BAN logic are described in Table 2.

To achieve mutual authentication, the following goals should be satisfied, as shown in Table 3.

The article "A Traceable Blockchain-Based Vaccination Record Storage and Sharing System" was published in 2022. Journal: J Healthc Eng.

The messages delivered between User A and User B are listed in Table 4.

To achieve the goals, the assumptions are made as shown in Table 5.

Based on the rules of BAN logic and these assumptions, the proof of the patient vaccination phase is as follows:

(a) User B authenticates User A.
    Statement *S*1 can be derived from *M*1 and the seeing rule.
   
*S*1. *B*⊲(〈*ID*_*A*_, *ID*_*B*_, *T*_1_〉_*PK*_*B*__, *r*_*A*_, *s*_*A*_)
    Statement *S*2 can be derived from *A*2 and the freshness rule.
   
*S*2. *B|* ≡ #(〈*ID*_*A*_, *ID*_*B*_, *T*_1_〉_*PK*_*B*__, *r*_*A*_, *s*_*A*_)
    Statement S3 can be derived from S1, A4, and the message meaning rule.
    S3. *B|* ≡ *A|* ~ (〈*ID*_*A*_, *ID*_*B*_, *T*_1_〉_*PK*_*B*__, *r*_*A*_, *s*_*A*_)
    Statement S4 can be derived from S2, S3, and the nonce verification rule.
    S4. *B|* ≡ *A|* ≡ (〈*ID*_*A*_, *ID*_*B*_, *T*_1_〉_*PK*_*B*__, *r*_*A*_, *s*_*A*_)
    Statement *S*5 can be derived from *S*4 and the belief rule.
   
*S*5 (*G*4) $B|\equiv Α\equiv Α\overset{x_{A}}{⟷}B$
    Statement *S*6 can be derived from *S*5, *A*6, and the jurisdiction rule.
   
*S*6 (G3) $B|\equiv A\overset{x_{A}}{⟷}B$
    Statement *S*7 can be derived from *S*3 and the belief rule.
   
*S*7 (*G*8) *B|*≡Α≡Ι*D*_*A*_
    Statement *S*8 can be derived from *S*7, *A*8, and the jurisdiction rule.
   
*S*8 (*G*7) *B|*≡Ι*D*_*A*_
(b) User A authenticates User B.
    Statement *S*9 can be derived from *M*2 and the seeing rule.
    S9. *A*⊲(〈*ID*_*B*_, *ID*_*A*_, *T*_2_〉_*PK*_*A*__, *r*_*B*_, *s*_*B*_)
    Statement S10 can be derived from A1 and the freshness rule.
    S10. *A|* ≡ #(〈*ID*_*B*_, *ID*_*A*_, *T*_2_〉_*PK*_*A*__, *r*_*B*_, *s*_*B*_)
    Statement S11 can be derived from S9, A3, and the message meaning rule.
    S11. *A|* ≡ *B|* ~ (〈*ID*_*B*_, *ID*_*A*_, *T*_2_〉_*PK*_*A*__, *r*_*B*_, *s*_*B*_)
    Statement S12 can be derived from S10, S11, and the nonce verification rule.
    S12. *A|* ≡ *B|* ≡ (〈*ID*_*B*_, *ID*_*A*_, *T*_2_〉_*PK*_*A*__, *r*_*B*_, *s*_*B*_)
    Statement S13 can be derived from S12 and the belief rule.
    S13 (G2) $A|\equiv B|\equiv B\overset{x_{B}}{⟷}A$
    Statement S14 can be derived from S13, A5, and the jurisdiction rule.
    S14 (G1) $A|\equiv B\overset{x_{B}}{⟷}A$
    Statement S15 can be derived from S12 and the belief rule.
    S15 (G6) *A|* ≡ *B|* ≡ *ID*_*B*_
    Statement S16 can be derived from S15, A7, and the jurisdiction rule.
    S16 (G5) *A|* ≡ *ID*_*B*_
    According to statements S6, S8, S14, and S16, these statements mutually authenticate the identities of User A and User B in the proposed scheme. Taking the patient vaccination phase into account, patient P and clinic C can authenticate each other through statements S17, S18, S19, and S20.
    S17 (G3) $C|\equiv P\overset{x_{P}}{⟷}C$
    S18 (G7) *C|* ≡ *ID*_*P*_
    S19 (G1) $P|\equiv C\overset{x_{C}}{⟷}P$
    S20 (G5) *P|* ≡ *ID*_*C*_

The article "A Traceable Blockchain-Based Vaccination Record Storage and Sharing System" was published in 2022. Journal: J Healthc Eng.

### 5.2. Nonrepudiation

To ensure the nonrepudiation in our proposed scheme, the message sent by the sender must be signed with the secret key of the sender. The receiver can verify the received message with the public key of the sender; therefore, the sender cannot deny sending the message.  Table 6 shows the verification equations that need to be verified by the receiver in every phase of the proposed scheme.

### 5.3. Data Integrity

To ensure the integrity of the message transmitted in each phase, this study applies the ECDSA to generate the signature value with the hash value. As shown in Algorithm 2, the signature *s* is generated by hash value *h*.  Table 7 lists the signatures in each phase. All the signatures need to be verified by the receiver, as shown in Table 6.

### 5.4. Resisting Replay Attack

The messages transmitted from the sender have added a sending timestamp and verified whether the timespan is valid in the receiver. The timestamp is added in each phase to resist the replay attack. For example, in the authentication phase, User A adds a timestamp *T*_1_ in the message *M*_*A*_, which will be encrypted by the public key of User B, as shown in equations (60) and (61). User B decrypts the cipher message and checks the validation of the timespan, as shown in equations (62) and (63). When a malicious attacker sends the same message to the receiver to achieve the replay attack, the receiver will decrypt the cipher message and compare the sending timestamp with the current time. If the timespan is larger than the threshold, the attack will fail. Therefore, the replay attack cannot succeed in our proposed scheme.

(60) $$\begin{array}{c} M_{A}=\left(ID_{A}||ID_{B}||T_{1}\right), \end{array}$$

(61) $$\begin{array}{c} C_{A}=E_{PK_{B}}\left(M_{A}\right), \end{array}$$

(62) $$\begin{array}{c} M_{A}=D_{SK_{B}}\left(C_{A}\right), \end{array}$$

(63) $$\begin{array}{c} \left(T_{2}-T_{1}\right)\leq \tau ?. \end{array}$$

### 5.5. Resisting Man-in-the-Middle Attack

In our method, the message sent by the sender is encrypted by the public key of the receiver. The receiver can decrypt the cipher message with its private key. When a malicious attacker intercepts the cipher message, he/she cannot decrypt without the relevant private key. Therefore, our proposed system can resist the man-in-the-middle attack.

## 6. Performance Analysis

We analyze the performance of our system in terms of the following aspects.

### 6.1. Computation Cost

The computation cost is also an important aspect to evaluate the performance of a system.  Table 8 elaborates the computation costs of our proposed scheme in each phase for BC, the hospital, the clinic, and the patient. It can be seen from Table 8 that each role has equal computation costs. For example, in the authentication phase, User A needs two symmetric encryption/decryption operations (*T*_*E*_), two hash function operations (*T*_*H*_), two additional operations (*T*_*A*_), one subtraction operation (*T*_*S*_), five multiplication operations (*T*_*M*_), and three division operations (*T*_*D*_).

The article "A Traceable Blockchain-Based Vaccination Record Storage and Sharing System" was published in 2022. Journal: J Healthc Eng.

### 6.2. Communication Cost

Assumed that an ID message required 128 bits, a cipher message required at least 512 bits, a signature message required 1024 bits, and other messages, like timestamp, requires 64 bits. As shown in the patient treatment phase, the patient encrypts the message, which contains 2 IDs, 1 timestamp, and a symptom described by the patient. The length of the symptom is set as 3 other messages, so the length of the cipher message is 2 × 128 bits +1 × 64 bits +3 × 64 bits = 512 bits.

Taking the patient treatment phase into account, the patient and the hospital will exchange 2 messages, which require 2 IDs, 1 cipher message, and 1 signature operation message. Thus, it requires (1282 + 5121 +  10241) 2 = 1792 bits in total. The maximum transmission speed is 14 Mbps, 100 Mbps, and 20 Gbps in a 3.5 G, 4G, and 5 G environment. Thus, the transmission time is only 0.015 ms, 0.002 ms, and 0.01 us, which reveals that our system can be utilized in various real-time applications.  Table 9 lists the communication costs of the proposed scheme in each phase.

### 6.3. Functionality Comparison

Table 10 shows the functionality comparison of previous schemes and the proposed scheme. Our proposed scheme has the advantage of providing theoretical proof, solving the nonrepudiation issue, and providing the man-in-the-middle attack resistance.

### 6.4. Limitations

There are some limitations in our system. First, every party must register in the blockchain center (BC) before joining the system. During the registration process, each participant needs to obtain the public key and private key pair of the elliptic curve signature from the BC. Second, the proposed scheme relies on stable power and network for normal operations. Thus, a backup power supply and a secure local network system can be established for the proposed system to prevent system failure.

Overall, the proposed scheme in this study is focused on applying blockchain technology to solve the storage and sharing for VR. Some potential problems are not comprehensively considered, for example, the unpopularity or slow speed of the internet environment.

The article "A Traceable Blockchain-Based Vaccination Record Storage and Sharing System" was published in 2022. Journal: J Healthc Eng.

## 7. Conclusions

This study discusses the problems that occurred in the application of the vaccination record (VR) in reality and proposes a blockchain-based vaccination record storage and sharing system. The integrity of the VR and the privacy protection problems are solved by using blockchain technologies. The security of our system was analyzed such as mutual authentication, nonrepudiation, and data integrity. Moreover, our method can resist replay attacks and man-in-the-middle attacks. In particular, we use BAN logic to prove identity legality such that communication security is guaranteed between two parties. Not merely the computational and communication costs are quite low, the proposed method can save time and avoid medical risks than the current medical system.

In the next work, we hope to improve the proposed system using artificial intelligence (AI) and deep learning techniques, which will be used to store VR in different formats and enable efficient VR search.

## Figures and Tables

**Figure 1:** The framework of the proposed system.

**Figure 2:** The primary information is defined in the smart contract.

**Figure 3:** The chaincode structure of the vaccination record is stored in BC.

**Figure 4:** The framework of the registration phase.

**Figure 5:** The flowchart of the authentication phase.

**Figure 6:** The flowchart of the patient vaccination phase.

**Figure 7:** The flowchart of the patient treatment phase.

**Algorithm 1:** The smart contract Registration

**Algorithm 2:** The smart contract Sign

**Algorithm 3:** The smart contract Verify

**Algorithm 4:** The algorithm RIns

**Algorithm 5:** The algorithm RGet.

**Table 1:** The notations used in this study.

Name	Description
*ID*_*X*_	The identity of *X*
*p*	A *k*-bit prime number
*F*_*p*_	Finite group of *p*
*E*	*E* the elliptic curve defined on finite group
*G*	*G* a generating point based on *E*
*R*_*i*_	The *i*-th random number based on *E*
(*r*_*X*_, *s*_*X*_)	The elliptic curve signature key pair for *X*
(*x*_*X*_, *y*_*X*_)	The ECDSA signature key pair for *X*
(*d*_*X*_, *Q*_*X*_)	(*d*_*X*_, *Q*_*X*_) the ECDSA private key and public key for *X*
*H*()	One-way hash function
(*SK*_*X*_, *PK*_*X*_)	The private key and public key for *X*
*C*_*X*_	The ciphertext send by *X*
*T*_*i*_	The *i*-th timestamp
*τ*	The threshold for checking the validity of timestamps
MX	The sending message from *X*
*E*_*PK*_*X*__(*M*)	Encrypt message *M* with the public key of *X*
*D*_*SK*_*X*__(*M*)	Decrypt message *M* with the private key of *X*
$X\overset{?}{=}Y$	Verify that *X* is equal to *Y* or not
*V*	The name of the vaccination
*S*	The symptom of the patient
*D*	The diagnostic result of the patient
VR	The vaccination record
*K*_*VR*_	The primary message of the VR

The article "A Traceable Blockchain-Based Vaccination Record Storage and Sharing System" was published in 2022. Journal: J Healthc Eng.

**Table 2:** Common notations are used in the BAN logic.

P *|*≡ X	P believes X

P ⊲ X	P sees X

P *|*∼*X*	P said X

P *|*⇒ X	P controls X

#(*X*)	X is fresh

$P\overset{K}{⟷}X$	P and *X* share the key K

$\overset{K}{⟶}P$	K is the public key of P

$P\overset{X}{⟺}Q$	P and *Q* share the secret X

**Table 3:** The goals of the authentication analysis.

*G*1	$A|\equiv B\overset{x_{B}}{⟷}A$

*G*2	$A|\equiv B|\equiv B\overset{x_{B}}{⟷}A$

*G*3	$B|\equiv A\overset{x_{A}}{⟷}B$

*G*4	$B|\equiv A|\equiv A\overset{x_{A}}{⟷}B$

*G*5	*A|* ≡ *ID*_*B*_

*G*6	*A|* ≡ *B|* ≡ *ID*_*B*_

*G*7	*B|* ≡ *ID*_*A*_

*G*8	*B|* ≡ *A|* ≡ *ID*_*A*_

**Table 4:** The delivered messages.

*M*1	*User* *A*⟶*User* *B*(〈*ID*_*A*_, *ID*_*B*_, *T*_1_〉_*PK*_*B*__, *r*_*A*_, *s*_*A*_)

*M*2	*User* *B*⟶*User* *A*(〈*ID*_*B*_, *ID*_*A*_, *T*_2_〉_*PK*_*A*__, *r*_*B*_, *s*_*B*_)

**Table 5:** The assumptions between User A and User B.

*A*1	*A|* ≡ #(*T*_1_)
*A*2	*B|* ≡ #(*T*_1_)

*A*3	*A|* ≡ #(*T*_3_)

*A*4	*B|* ≡ #(*T*_3_)

*A*5	$A|\equiv B|\equiv B\overset{x_{B}}{⟷}A$

*A*6	$B|\equiv A|\equiv A\overset{r_{A}}{⟷}B$

*A*7	*A|* ≡ *B|*⟹*ID*_*B*_

*A*8	*B|* ≡ *A|*⟹*ID*_*A*_

**Table 6:** Nonrepudiation of the proposed scheme.

Phases	Items		
	Sender	Receiver	Verification
Authentication phase	User A	User B	*Verify*(*h*_*A*_′, *r*_*A*_, *s*_*A*_)
	User B	User A	*Verify*(*h*_*B*_′, *r*_*B*_, *s*_*B*_)
Patient vaccination	Patient	Clinic	*Verify*(*h*_*P*_′, *r*_*P*_, *s*_*P*_)
	Clinic	Patient	*Verify*(*h*_*C*_′, *r*_*C*_, *s*_*C*_)
Patient treatment	Patient	Hospital	*Verify*(*h*_*P*2_′, *r*_*P*2_, *s*_*P*2_)
	Hospital	Patient	*Verify*(*h*_*H*_′, *r*_*H*_, *s*_*H*_)

**Table 7:** Data integrity of the proposed scheme.

Phases	Items		
	Sender	Receiver	Signature
Authentication phase	User A	User B	(*r*_*A*_, *s*_*A*_)=*Sign*(*h*_*A*_, *R*_1_, *d*_*A*_)
	User B	User A	(*r*_*B*_, *s*_*B*_)=*Sign*(*h*_*B*_, *R*_2_, *d*_*B*_)
Patient vaccination	Patient	Clinic	(*r*_*P*_, *s*_*P*_)=*Sign*(*h*_*P*_, *R*_3_, *d*_*P*_)
	Clinic	Patient	(*r*_*C*_, *s*_*C*_)=*Sign*(*h*_*C*_, *R*_4_, *d*_*C*_)
Patient treatment	Patient	Hospital	(*r*_*P*2_, *s*_*P*2_)=*Sign*(*h*_*P*2_, *R*_5_, *d*_*P*2_)
	Hospital	Patient	(*r*_*H*_, *s*_*H*_)=*Sign*(*h*_*H*_, *R*_6_, *d*_*H*_)

**Table 8:** The computation costs of the proposed scheme.

Phase	Role 1	Role 2
Authentication	User A:	User B:
	2*T*_*E*_ *+* 2*T*_*H*_ *+* 2*T*_*A*_ *+* *T*_*S*_ *+* 4*T*_*M*_ *+* 3*T*_*D*_	2*T*_*E*_ *+* 2*T*_*H*_ *+* 2*T*_*A*_ *+* *T*_*S*_ *+* 4*T*_*M*_ *+* 3*T*_*D*_
Patient vaccination	Patient:	Clinic:
	2*T*_*E*_ *+* 2*T*_*H*_ *+* 2*T*_*A*_ *+* *T*_*S*_ *+* 4*T*_*M*_ *+* 3*T*_*D*_	2*T*_*E*_ *+* 2*T*_*H*_ *+* 2*T*_*A*_ *+* *T*_*S*_ *+* 4*T*_*M*_ *+* 3*T*_*D*_
Patient treatment	Patient:	Hospital:
	2*T*_*E*_ *+* 2*T*_*H*_ *+* 2*T*_*A*_ *+* *T*_*S*_ *+* 4*T*_*M*_ *+* 3*T*_*D*_	2*T*_*E*_ *+* 2*T*_*H*_ *+* 2*T*_*A*_ *+* *T*_*S*_ *+* 4*T*_*M*_ *+* 3*T*_*D*_

The article "A Traceable Blockchain-Based Vaccination Record Storage and Sharing System" was published in 2022. Journal: J Healthc Eng.

**Table 9:** The communication costs of the proposed scheme.

Phase	Message length (bits)	3.5 *G* (ms)	4 *G* (ms)	5 *G*
Authentication	1792	0.015	0.002	0.01 *us*
Patient vaccination	1792	0.015	0.002	0.01 *us*
Patient treatment	1792	0.015	0.002	0.01 *us*

**Table 10:** The functionality comparison of previous schemes and the proposed scheme.

Scheme functionality	Xu et al. [17]	Liu et al. [22]	Xu et al. [23]	Our scheme
Internet of things (IoTs)	Yes	No	No	No
Blockchain architecture	No	Yes	Yes	Yes
Mutual authentication	No	Yes	Yes	Yes
Data integrity	Yes	Yes	Yes	Yes
Resistance to replay attack	No	Yes	Yes	Yes
Resistance to man-in-the-middle attack	No	No	No	Yes
Nonrepudiation	No	No	Yes	Yes
Theoretical proof	No	No	No	Yes

## Data Availability

The data supporting this study are available within the article.
